The article "Thoracic Paravertebral Nerve Block with Ropivacaine and Adjuvant Dexmedetomidine Produced Longer Analgesia in Patients Undergoing Video-Assisted Thoracoscopic Lobectomy: A Randomized Trial" was published in 2021. Journal: J Healthc Eng.

# Thoracic Paravertebral Nerve Block with Ropivacaine and Adjuvant Dexmedetomidine Produced Longer Analgesia in Patients Undergoing Video-Assisted Thoracoscopic Lobectomy: A Randomized Trial

**DOI:** 10.1155/2021/1846886

**Published:** 2021-09-08

**Authors:** Jun Zha, Shiliang Ji, Chen Wang, Zhe Yang, Shigang Qiao, Jianzhong An

**Affiliations:** ^1^Department of Anesthesiology and Perioperative Medicine, The Affiliated Suzhou Science & Technology Town Hospital of Nanjing Medical University, No. 1 Lijiang Road, Suzhou 215153, China; ^2^Department of Pharmacy, The Affiliated Suzhou Science & Technology Town Hospital of Nanjing Medical University, No. 1 Lijiang Road, Suzhou 215153, China; ^3^Institute of Clinical Medicine Research, The Affiliated Suzhou Science & Technology Town Hospital of Nanjing Medical University, No. 1 Lijiang Road, Suzhou 215153, China

## Abstract

**Purpose:**

This study evaluated the postoperative analgesic effect of ultrasound-guided single-point thoracic paravertebral nerve block (TPVB) combined with dexmedetomidine (DEX) in patients undergoing video-assisted thoracoscopic lobectomy.

**Methods:**

Sixty adult patients of the American Society of Anesthesiologists (ASA) I–III were randomly assigned into three groups (*n* = 20 each). G group: patients received routine general anesthesia; PR group: patients received 0.5% ropivacaine; and PRD group: patients received 0.5% ropivacaine with 1 *μ*g/kg DEX. TPVB was performed in the T5 space before surgery, and then, general anesthesia induction and video-assisted thoracoscopic lobectomy were performed. Analgesics were administered through the patient-controlled analgesia (PCA) device intravenously. The background infusion of each PCA device was set to administer 0.02 *μ*g/kg/h sufentanil, with a lockout time of 15 min, and a total allowable volume is 100 ml.

**Results:**

Compared to PR and G groups, the total sufentanil consumption after operation, the times of analgesic pump pressing, the pain score, and the incidence of postoperative nausea or vomiting in the PRD group were significantly reduced (*p* < 0.05). Also, the duration of first time of usage of the patient-controlled analgesia (PCA) was longer. The heart rate (HR) and mean arterial pressure (MAP) during operation were lower in the PRD group as compared with the other two groups in most of the time. However, hypotension and arrhythmia occurred in three groups with no statistically significant difference.

**Conclusions:**

A small volume of TPVB with ropivacaine and DEX by single injection produced longer analgesia in patients undergoing video-assisted thoracoscopic lobectomy, reduced postoperative opioids consumption, and the incidence of side effects.

The article "Thoracic Paravertebral Nerve Block with Ropivacaine and Adjuvant Dexmedetomidine Produced Longer Analgesia in Patients Undergoing Video-Assisted Thoracoscopic Lobectomy: A Randomized Trial" was published in 2021. Journal: J Healthc Eng.

## 1. Introduction

Video-assisted thoracoscopic surgery (VATS) is mainly used for the treatment of the lung, mediastinum, and pleural lesions. The main advantage is to avoid the injury of thoracotomy. Compared with thoracotomy, the operation time is shorter, the postoperative morbidity is lower, and the time for returning to normal activities is earlier [1]. However, effective analgesia is still needed to reduce postoperative pain and postoperative nausea and vomiting.

Thoracic paravertebral block (TPVB) as part of a multimodal analgesia strategy after thoracotomy [2] and breast surgery [3] has a broad evidence base and along with ultrasound-guided techniques. It has become increasingly popular. Recent randomized controlled trials and reviews have shown that paravertebral block (PVB) causes prolonged directional analgesia and reduces the risk of postoperative nausea, vomiting, and complications [4, 5]. However, a large body of literature has shown that the duration of analgesia is controversial, and PVB is only beneficial immediately after surgery [6, 7]. There are few studies on the effectiveness and tolerability of adjuvant analgesics in paraspinal analgesia. The addition of magnesium, clonidine, ketamine, dexamethasone, opioids, and other analgesics and local anesthetics can enhance and prolong the analgesic effect provided by PVB [8, 9].

Dexmedetomidine (DEX) is a novel alpha-2 adrenergic receptor agonist with dose-dependent sedative, anxiolytic, and analgesic effects and has an advantage of minimum respiratory depression compared with alternative drugs [10]. It is well known that *α*-_2_ receptor agonists, due to their own sympathetic properties, provide stable hemodynamics during surgery and reduce the amount of narcotic analgesics. When DEX is used as an anesthetic for epidural anesthesia [11], subarachnoid block [12, 13], PVB [14, 15], and brachial plexus block analgesia [16], the time is significantly extended. However, there are few studies evaluating the efficacy of DEX as an adjuvant in the treatment of analgesia after thoracoscopic surgery, only in partial breast surgery [15].

Therefore, this study was designed to evaluate whether TPVB combined with ropivacaine and DEX could improve the analgesic effect of patients undergoing VATS, thereby reducing postoperative opioid drugs consumption.

## 2. Methods

This study was approved by the Affiliated Suzhou Science and Technology Town Hospital of Nanjing Medical University' Ethics Committee, and written informed consent was obtained from all patients. The trial is registered at the Chinese Clinical Trial Registry, number ChiCTR-IOR-17013034. After obtaining approval and written informed consent from the institutional ethics committee, the study enrolled 60 ASA I–III patients (18–65 years old, either gender, weighing 50–85 kg) who were scheduled to undergo elective thoracoscopic lobectomy. Patients undergoing elective general anesthesia and video-assisted thoracoscopic unilateral lobectomy had no history of cardiopulmonary disease, no sinus bradycardia, no functional lesions of the sinoatrial node, no serious arrhythmia, and no thoracic deformity. Surgery time was more than 2 hours. Exclusion criteria: minimental state examination scores below 23 points; the history of dementia, psychosis, or other central nervous system disease or drug dependence and poor compliance; and those who did not complete video-assisted thoracoscopic lobectomy under general anesthesia or have to convert to thoracotomy.

The article "Thoracic Paravertebral Nerve Block with Ropivacaine and Adjuvant Dexmedetomidine Produced Longer Analgesia in Patients Undergoing Video-Assisted Thoracoscopic Lobectomy: A Randomized Trial" was published in 2021. Journal: J Healthc Eng.

All patients did not use preoperative medication, and in the preoperative preparation room, the patients were explained in detail the numerical rating scale (NRS) scoring rules (scores from 0 to 10: 0 = no pain, 10 = most severe pain). Patients were randomized into three groups of 20 individuals each using a computer-generated random number table (random number table method) with sealed envelope technology for assignment concealment (distribution hidden). In the operating room, ultrasound-guided right internal jugular vein catheterization for infusion and left radial artery catheterization for monitoring the changes of pressure have been performed. Conventional general anesthesia induction included sufentanil 5 ug/kg + etomidate 2 mg/kg + cisatracurium 2 mg/kg intravenous slow bolus injection; anesthesia maintenance: propofol 2.5 ug/ml, sevoflurane 0.8 MAC, remifentanil 3 ng/ml, bispectral index monitoring, and the depth of anesthesia is maintained between 40 and 60. Patients were classified into three groups as follows: G group: patients received routine general anesthesia; PR group: patients received 0.5% ropivacaine for TPVB; PRD group: patients received 0.5% ropivacaine with 1 *μ*g/kg DEX for TPVB. Paravertebral blockade was performed under ultrasound guidance. A linear ultrasound transducer (HITACHI Arietta 60) was placed intercostally to identify the thoracic paravertebral space (TPVS), and a 20-gauge needle was inserted into the plane of the transducer. When the needle tip reached TPVS, 10 mL 0.5% ropivacaine with 1 *μ*g/kg DEX in T5 paravertebral space was injected.

The gender, age, ASA grade, height, weight, body mass index (BMI), heart rate (HR), mean artery pressure (MAP) baseline, duration of surgery (h), anesthesia (h), the time to first analgesic request since paravertebral injection (TFR1), first use of patient-controlled analgesia (PCA1) intravenously, total sufentanil dosage, and the pressing times of analgesic pumps were all recorded in three groups. The intraoperative MAP and HR were measured after starting TPVB bolus injection. Hypotension defined as a 30% decrease or less than 80 mmHg in systolic blood pressure from baseline was treated with ephedrine 5 mg intravenously and further boluses as required. Bradycardia defined as heart rate <55 beats per minute was treated with 0.6 mg intravenously. Analgesics were administered through the PCA device (ZZB-150, Apon, Nantong, China). The background infusion of each PCA device was set to administer 0.02 *μ*g/kg/h sufentanil, with a lockout time of 15 min, and a total allowable volume is 100 ml. The anesthetist conducted postoperative monitoring, pain assessment, and management was blinded to the patient groups. The flowchart of the study protocol is shown in Figure 1.

The article "Thoracic Paravertebral Nerve Block with Ropivacaine and Adjuvant Dexmedetomidine Produced Longer Analgesia in Patients Undergoing Video-Assisted Thoracoscopic Lobectomy: A Randomized Trial" was published in 2021. Journal: J Healthc Eng.

Ramsay sedation scores of patients were recorded at 30 minutes, 1 hour, 2 hours, 4 hour, 6 hours, 8 hours, 12 hours, and 24 hours after anesthetic recovery in three groups (score 1: patient anxiety, agitated or restlessness, or both; score 2: patient cooperation, orientation, and calm; score 3: patient only responds to orders; score 4: patient with light outer membrane percussion, or a loud auditory stimuli showed a rapid response; score 5: the patient showed a slow response to light eyebrows or loud auditory stimuli; score 6: the patient did not respond; score 2–4 is an ideal sedation level). The intraoperative MAP and HR were recorded at 10 minutes, 20 min, 30 min, 40 min, 50 min, 60 min, 70 min, 80 min, 90 min, and 100 min after starting TPVB bolus injection. Postoperative pain ratings (NRS) during rest and movement were recorded every two hours within 24 hours (NRS: NRS uses 0–10 to represent different degrees of pain. Score 0: no pain; score 1–3: mild pain; score 4–6: moderate pain; score 7–10: severe pain).

All values are mean ± SEM. Two-way ANOVA for repeated measures was used when appropriate (SPSS 20.0 for Windows, SPSS Inc.). The Student–Newman–Keuls multiple comparison post hoc test was used to differentiate within the groups. A probability value less than 0.05 was considered to indicate a significant difference between the groups, while a value greater than 0.05 was considered to indicate no significant difference between the groups.

## 3. Results

There were no significant differences among the G group, PR group, and PRD group in demographic data such as age, weight, height, BMI, and baseline hemodynamic parameters durations of surgery and anesthesia (*p* > 0.05) (Table 1). All patients underwent the surgery successfully without local anesthetic toxicity or diclofenac sodium contraindications.

The article "Thoracic Paravertebral Nerve Block with Ropivacaine and Adjuvant Dexmedetomidine Produced Longer Analgesia in Patients Undergoing Video-Assisted Thoracoscopic Lobectomy: A Randomized Trial" was published in 2021. Journal: J Healthc Eng.

Postoperative sufentanil (over 24 hours) consumptions were reduced significantly in the PRD group compared to other two groups (*p* < 0.05; Table 2). Moreover, all the abovementioned parameters did not reach significant difference between the G group and PR group as given in Table 2 (*p* > 0.05). There was no significant difference of postoperative Ramsay sedation scores among all groups before 12 h; however, the score values in the G group were significantly lower than that in the PR or PRD group (*p* < 0.05; Table 3).

The NRS pain scores of ipsilateral arm were, respectively, indicated in Figure 2 and 3 in rest or movement status. There was no significant difference in pain score among three groups in rest or movement status within 1 hour after surgery; 2 hours after surgery, the pain scores of the PRD group were lower than other two groups. In the PRD group, TFR1 and PCA1 were significantly longer than those in the PR group (*p* < 0.05) and G group (*p* < 0.05) (Table 2). There were significant differences of TFR1 and PCA1 between the PR group and *G* group (*p* < 0.05).

Hemodynamic parameters were monitored during surgery. HR and MAP trends are shown in Figures 4 and 5, respectively. There were no differences of hypotension and bradycardia among groups and the requirement of vasopressors for maintenance of stable hemodynamic parameters during the induction period did not show significant differences among groups (data not shown). The intraoperative HR and MAP in the PRD group were lower compared to other two groups. After 10 minutes, the intraoperative HR of all three groups decreased, but it was more obvious in the PR group and G group than that in the PRD group (*p* < 0.05). In the PR group and G group, the intraoperative HR tended to stabilize and increased slowly until 40 minutes, but the HR of the PRD group was lower than other G groups at 80 and 100 minutes. In the PR group and G group, the intraoperative MAP decreased significantly around 20 minutes, while MAP of the PRD group decreased to (77.1 ± 1.7) mmHg around 40 minutes, and it gradually returned to the baseline level around 100 minutes (*p* < 0.05). However, there was no significant difference in the consumption of sufentanil dose or the incidence of hypotension and the occurrence of bradycardia during the surgery.

## 4. Discussion

TPVB has been used wildly to reduce postoperative opioid consumption and provide effective pain control. The injection site and volume are quite different in different studies, and there are single and multiple injections with volumes of 5, 7, 10, 15, 20, or 0.3 ml/kg [17]. A cadaver study observed distribution of 20 ml injected dye over three to four TPVS (range, 1–10) with 40% incidence of epidural spread [2]. Therefore, the analgesic effect produced by the volume of 15 or 20 ml may also include the effect of the epidural spread. In this study, we applied a volume of 10 ml of DEX combined with ropivacaine TPVB for patients with thoracoscopic lobectomy had a better analgesic effect than patients with only TPVB or no TPVB and may reduce the incidence of epidural spread.

The article "Thoracic Paravertebral Nerve Block with Ropivacaine and Adjuvant Dexmedetomidine Produced Longer Analgesia in Patients Undergoing Video-Assisted Thoracoscopic Lobectomy: A Randomized Trial" was published in 2021. Journal: J Healthc Eng.

DEX acts as a potential adjuvant for both axons and peripheral nerve blocks [16, 18], and studies have confirmed that epidural injection of DEX enhanced local anesthetics on nerves, reduced the need for intraoperative anesthesia, and provided a better analgesic effect after thoracotomy [19]. The analgesic effect is concentrated by inhibiting the release of substance P in the nociceptive pathway of dorsal root neurons and activating the alpha-2 receptor in the blue spot. This alpha-2 agonist mediates peripheral analgesia by reducing the release of norepinephrine and the independent inhibition of neurofibrillary action potential by the alpha-2 receptor. None of the various animal studies showed any adverse neurological effects of DEX [20, 21] and neuroprotective effects of dexmedetomidine, induced by intrathecal administration is similar to methylprednisolone [21]. DEX has also been used in human studies as an adjuvant for local anesthetics [14, 15]. Mahendru et al. compared the effects of intrathecal DEX and fentanil as bupivacaine adjuvants; the results showed that intrathecal DEX prolonged exercise and sensory block, more hemodynamic stability, and reduced need for analgesics within 24 hours compared with fentanil [22]. In other studies, DEX improved blocker efficiencies have been shown, with no reported neurological side effects. Further study of the neuronal effects of DEX was encouraged by the researchers [15, 16]. In the current study, the consumption of sufentanil in the two paravertebral nerve block patients was significantly lower than that in the control group, indicating that paravertebral nerve block can prolong the analgesic time. None of the patients in the PRD group required an additional dose of sufentanil, while only one patient in the PR group required an additional dose of sufentanil. Compared with the PR group and the G group, the first analgesia request time was much longer in the PRD group, and the postoperative PRD group had a longer PCA1 time, but the total number of PCA (or sufentanil consumption) and pain score are lower. This indicates that ropivacaine supplemented with DEX prolongs the time of analgesia after PVB. In addition, patients receiving DEX had less opioid-related complications such as nausea and vomiting. On the other hand, all of these parameters were comparable in the PR group and G group, indicating that there was no significant TPVB analgesic effect of ropivacaine alone compared with patients who did not receive TPVB. The use of local anesthetic TPVB alone improved intraoperative analgesia and reduced the need for sufentanil, but did not provide adequate postoperative analgesia. A recent RCT meta-analysis study evaluated the analgesic effects of multilevel TPVB in combination with ropivacaine or bupivacaine in postoperative breast cancer [23], and the results showed the overall analgesic consumption was lower in the intraoperative and postoperative ropivacaine groups or bupivacaine group, and the number of patients with NRS >3 after PACU was significantly reduced in the TPVB group. The local anesthetic infiltration group immediately reduced postoperative pain, especially in the 2 hours after surgery, but there was no significant difference of analgesia between 12 hours and 24 hours after surgery.

The article "Thoracic Paravertebral Nerve Block with Ropivacaine and Adjuvant Dexmedetomidine Produced Longer Analgesia in Patients Undergoing Video-Assisted Thoracoscopic Lobectomy: A Randomized Trial" was published in 2021. Journal: J Healthc Eng.

In this study, the requirement of vasopressors for maintenance of stable hemodynamic parameters did not reveal any significant difference during the induction period among groups. However, the HR and MAP in the PRD group were lower than those in the other two groups during surgery. It has been reported that the stable hemodynamics may possibly be explained on the basis of lower volume of local anesthetics used and a suitable selection of the dose of adjuvant [11]. The sedative effects found in the study may be related to the use of DEX [24]. A higher sedation score in the PR and PRD groups than the G group may due to better analgesia effects in PR and PRD groups.

More recently, Hong et al. reported that DEX as an adjunct in TPVB provided effective pain relief and significantly reduced opioid requirement in VATS [25]. Our results are consistent with the Hong et al.' study. However, there are two differences between our study and Hong et al. study'. (1) In our study, only on injection at T5 space before surgery, while there are two injections at the T3-T4 and T4-T5 levels after surgery in Hong et al.' study. It has been reported that TPVB performed prior to general anesthesia for laparoscopic cholecystectomy can provide early discharge and better postoperative pain management [6]. (2) The injection volume of the ropivacaine and DEX is different. The injection volume of ropivacaine and DEX mixture in our study is 10 ml at the single site, while the total volume of the two site injections was 30 ml in Hong et al.' study. Our results demonstrated that a small injection volume (10 ml 0.5% ropivacaine with 1 *μ*g/kg DEX) at site of T5 space before surgery also achieved effective postoperative analgesia. It may have beneficial clinical effects for reducing the side effects of drugs, puncture injury, and discomfort to patients and enhancing recovery after surgery.

The article "Thoracic Paravertebral Nerve Block with Ropivacaine and Adjuvant Dexmedetomidine Produced Longer Analgesia in Patients Undergoing Video-Assisted Thoracoscopic Lobectomy: A Randomized Trial" was published in 2021. Journal: J Healthc Eng.

There are certain limitations to our study. First, it was a retrospective study with a small sample size and the findings therefore have to be confirmed with a larger randomized controlled trial. Second, the small sample size and recruitment of relatively healthy patients (ASA I and II) limited the possibility of drawing a definitive conclusion. Greater numbers of patients and patients with multiple comorbidities (i.e., ASA III or IV) need to be included in future studies to verify these findings. Third, since a single dose of TPVB can provide sufficient pain relief, inserting a catheter into the paravertebral space for continuous infusion of local anesthetics may provide protracted postsurgery analgesia. Furthermore, different doses and drugs used in TPVB may cause bias of the results. More studies have to be conducted to clarify this question.

## 5. Conclusions

In summary, a small volume of TPVB with 1 *μ*g/kg DEX combined with 0.5% ropivacaine by single injection at T5 space before surgery for patients undergoing thoracoscopic lobectomy prolonged the overall analgesia time after surgery and reduced the dose and side effects of opioids.

## Figures and Tables

**Figure 1:** CONSORT flow diagram of the study.

**Figure 2:** Postoperative NRS.R. Values in all groups. Values in the PRD group compared to the G group and the PR group at all time points. There was no difference between the G group and PR group (*p* > 0.05).

**Figure 3:** Postoperative NRS.M. Values in all groups. Values in the PRD group compared to the G group and the PR group at all time points (*p* < 0.05). There was no difference between the G group and PR group.

**Figure 4:** Intraoperative heart rate values in all groups. The PRD group compared to the G group and PR group except at 40 minutes and 60 minutes (^*∗*^*p* < 0.05).

**Figure 5:** Intraoperative MAP values in all groups. The PRD group compared to the G group and PR group except at 20 min and 100 min (^*∗*^*p* < 0.05). There were significant differences between the G group and PR group at 60, 80, and then 100 min; the G group and PRD group at all time points except 20 min; and the PR group and PRD group at 20 and 100 min (*p* < 0.05).

**Table 1:** Characteristics of the patients and surgery.

Items	G group (*n* = 20)	PR group (*n* = 20)	PRD group (*n* = 20)	*P* value
Age (years)	45.7 ± 1.3	47.1 ± 1.7	48.1 ± 1.5	0.962
Height (cm)	165.4 ± 1.4	165.9 ± 1.2	164.6 ± 1.4	0.594
Weight (kg)	68.0 ± 2.1	67.3 ± 2.3	72.4 ± 2.1	0.719
BMI (kg/m^2^)	23.2 ± 0.5	23.4 ± 0.6	24.1 ± 0.6	0.574
Baseline HR (beats/min)	83.0 ± 1.6	82.3 ± 2.9	84.8 ± 2.3	0.922
Baseline MAP (mmHg)	96.7 ± 1.8	97.1 ± 1.5	95.5 ± 1.9	0.460
Surgery time (h)	2.2 ± 0.1	2.2 ± 0.1	2.2 ± 0.1	0.614
Anesthesia time (h)	2.5 ± 0.1	2.8 ± 0.1	2.9 ± 0.1	0.067

Values are mean ± SEM. G: general anesthesia; PR, paravertebral ropivacaine; PRD, paravertebral ropivacaine and dexmedetomidine; BMI, body mass index; HR, heart rate; MAP, mean arterial pressure.

The article "Thoracic Paravertebral Nerve Block with Ropivacaine and Adjuvant Dexmedetomidine Produced Longer Analgesia in Patients Undergoing Video-Assisted Thoracoscopic Lobectomy: A Randomized Trial" was published in 2021. Journal: J Healthc Eng.

**Table 2:** Analgesic efficacy and postoperative adverse effects.

Items	G group (*n* = 20)	PR group (*n* = 20)	PRD group (*n* = 20)	*P* value
TFR1 (h)	2.6 ± 1.5	5.6 ± 2.0	24.1 ± 2.9	<0.05^*∗*#$^
Numbers of pressing analgesic pump	5.3 ± 0.2	3.2 ± 0.1	1.6 ± 0.2	<0.05^*∗*#$^
Total sufentanil dosage (*μ*g)	142.2 ± 7.3	105.1 ± 5.7	78.2 ± 6.2	<0.05^*∗*#$^
Nausea	5(25%)	3(15%)	0	<0.05^*∗*#$^
Vomiting	2(10%)	1(5%)	0	<0.05^*∗*#$^

Values are mean ± SEM or *n* (%). TFR1, time from paravertebral injection to first analgesic request. *P* < 0.05, ^*∗*^G group vs. PR group; ^#^G group vs. PRD group; ^$^PR group vs. PRD group.

**Table 3:** Postoperative Ramsay sedation scores at different intervals.

Time points	G group (*n* = 20)	PR group (*n* = 20)	PRD group (*n* = 20)	*P* value
30 min	2.5 (2.0–5.0)	2.5 (2.0–5.0)	2.0 (2.0–5.0)	0.409
1 h	2.0 (2.0–4.0)	2.0 (2.0–4.0)	2.0 (2.0–4.0)	0.995
2 h	2.0 (2.0–4.0)	2.0 (2.0–4.0)	2.0 (2.0–4.0)	1.000
4 h	2.0 (2.0-3.0)	2.0 (2.0-3.0)	2.0 (2.0-3.0)	0.415
8 h	2.0 (2.0-3.0)	2.0 (2.0-3.0)	2.0 (2.0-3.0)	0.216
12 h	2.0 (2.0-3.0)	2.0 (2.0-3.0)	2.0 (2.0-3.0)	0.331
24 h	1.0 (0.0–2.0)	2.0 (1.0–3.0)	2.0 (0.0–3.0)	<0.05^*∗*#^

Values as median (interquartile range). ^*∗*^G group versus PR group; ^#^G group versus PRD group.

## Data Availability

The data used to support the findings of this study are available from the corresponding author upon request.
